This article has been retracted.

# Evaluating the influence of characteristics on the acceptance of artificial intelligence application: An empirical study

**DOI:** 10.1016/j.heliyon.2024.e39460

**Published:** 2024-10-17

**Authors:** Athapol Ruangkanjanases, Ornlatcha Sivarak, Chin-Tsu Chen, Asif Khan, Shih-Chih Chen

**Affiliations:** a Chulalongkorn Business School, Chulalongkorn University, Bangkok, Thailand; b Mahidol University International College, Mahidol University, Nakhon Pathom, Thailand; c Department of Commercial Design and Management, National Taipei University of Business, Taipei, Taiwan; d College of Business, Southern Taiwan University of Science and Technology, Tainan, Taiwan; e Department of Information Management, College of Management, National Kaohsiung University of Science and Technology, Kaohsiung, Taiwan

**Keywords:** Artificial intelligence, Interactivity characteristics, Richness characteristics, Reliability characteristics, Personalized characteristics, Map APP, User trust, User satisfaction, Continuance intention

## Abstract

Artificial intelligence has accelerated the application scenarios and business value of map applications. However, the sustained intention of map applications utilizing artificial intelligence technology has not received sufficient attention and scholarly investigation. Therefore, this study constructs a theoretical model of the continuance intention of map applications, based on their characteristics and combined with user satisfaction and trust, aiming to explore the influence mechanism of this continuance intention. The results of structural equation modeling show that not only user trust and satisfaction have a positive effect on continuance intention towards map applications, but also interactivity characteristics, reliability characteristics, richness characteristics, and personalized characteristics have a positive effect on user satisfaction and trust towards map applications. This study reveals the influence mechanism of map application continuance intention, which can effectively guide map application operators to optimize their services and then provide practical insights for users to use map applications consistently.

## 1 Introduction

With the development of information technology and the Internet, artificial intelligence (AI) technology is becoming increasingly mature and gradually applied in traffic, transportation, storage, and finance; the residents' needs for going out and entertainment have increased significantly compared with the past. As one of the high-tech products, smartphones are widely used to bring great convenience for residents to go out to work, shop, and travel. The growing travel demand of the population is driving the rapid growth of user access to geographic data information, leading to the growing popularity of map app applications [1,2]. The mobile mapping market has reached maturity, and mobile mapping APPs are tools with high homogeneity, i.e., once users install one mapping software, they generally do not install another mapping software, and competition among mapping software operators is intense [3,4]. It has been shown that the identification and development of user needs by R&D staff can effectively improve product market competitiveness and performance [5]. Undoubtedly, software operators need to meet the needs of map app users and promote their continued use. User intention to use refers to the likelihood that users are willing to use a product or technology, which can be divided into the initial intention to use and continuance intention based on the number of uses [6,7]. In this study, in the context of map app usage, continuance intention is the tendency of users to be willing to continue using a map APP after using it for the first time. Currently, academics are more concerned with the study of APP continuance intention [8].

AI has significantly transformed numerous sectors, with map applications being a prominent example. AI has augmented the functionality of these applications by incorporating advanced features such as real-time traffic updates, predictive routing, and tailored recommendations [9]. These innovations have not only increased the practicality of map applications but have also enhanced the overall user experience [10]. Essential characteristics such as interactivity [11], richness [12], reliability [13], and personalization [14] have emerged as key factors affecting user satisfaction and trust. Interactivity elements, like real-time feedback and adaptive interfaces, engage users more effectively and make the applications more responsive to their needs [15,16]. Richness attributes, which include the breadth and depth of information available, provide users with detailed and contextually relevant data, thus boosting satisfaction. Reliability, defined by the precision and consistency of information, is vital for establishing user trust, as users rely on these applications for accurate navigation and decision-making [5]. Personalized features, which customize the application experience based on individual user preferences, further enhance satisfaction and trust by offering a user-focused service [17]. However, the long-term intention of users to continue using AI-enhanced map applications has not been thoroughly examined. This study aims to fill this gap by exploring how these characteristics—interactivity, richness, reliability, and personalization—impact user satisfaction and trust, and consequently, the intention to continue using map applications.

Studies have classified users' perceived service characteristics of mobile apps into three dimensions: work compatibility, information usefulness, and communication correspondence, and explored their effects on users' attitudes and continuance intention using apps [18]. Lee et al. [19] used a structural model to investigate the relationship between service quality and post-use satisfaction, trust, immersion, and intention to use the fitness app again. Beldad & Hegner [20] explored the factors influencing the continued use of fitness apps by expanding the technology acceptance model (introducing social influence, trust, and health assessment). Yang et al. [21] studied users' persistent use behavior and its mechanism of action in social media contexts based on rooting theory, explaining that social attachment is the main factor leading to users' persistent intention. Studies have classified users' perceived service characteristics of mobile apps into three dimensions: work compatibility, information usefulness, and communication correspondence, and explored their effects on users' attitudes and continuance intention using apps [18]. Lee et al. [19] used a structural model to investigate the relationship between service quality and post-use satisfaction, trust, immersion, and continuance intention to use the fitness app again. Beldad & Hegner [20] explored the factors influencing the continuance intention of fitness apps by expanding the technology acceptance model (introducing social influence, trust, and health assessment). Academic research on the continuance intention of apps is more enthusiastic. From the research objects of the existing literature, academic studies on app continuance intention, such as knowledge payment, short video, psychology, and fitness, have been discussed [6,22,23], but studies on map and travel navigation apps are more limited. From the research content, the existing scholars' research on mobile app continuance intention is mostly based on improving existing theoretical models, users' online reviews, and the perceived characteristics of their use to construct app continuance intention models, and few scholars study the app characteristics as the starting point of its continuance intention [24,25]. More importantly, many scholarly studies have found that continuance intention is influenced by satisfaction and trust [21,[26], [27], [28], [29]].

Previous studies have underscored the critical role of satisfaction and trust in shaping continuance intention across various digital platforms [28,30]. Nevertheless, there is a noticeable lack of research that delves into how these factors interact specifically within the realm of AI-powered map applications. This research seeks to fill this gap by developing a theoretical framework that combines these characteristics with satisfaction and trust. Furthermore, aims to uncover the fundamental processes that influence users' intentions to continue using these applications. The central research question posed by this study is: In what ways do the interactivity, richness, reliability, and personalization features of AI-driven map applications affect user satisfaction and trust, and how do these elements subsequently impact continuance intention? Exploring this question will yield critical insights for developers and operators of map applications, helping them enhance their offerings and encourage sustained user engagement. In summary, considering the importance of users' usage needs and usage behaviors to map APP operators, this study combines the existing literature with the characteristics of map APP as an entry point to explore whether map APP users have continuance intention for the software because of trust or satisfaction in the context of artificial intelligence, to analyze the influence mechanism of map APP continuance intention. Moreover, based on the theoretical model and hypothesis testing results, this study provides corresponding practical insights for software operators to maintain users and improve their continuance intention.

## 2 Literature review and hypotheses development

### 2.1 Background

The incorporation of AI into map applications has dramatically enhanced the user experience, introducing functionalities that were previously beyond reach. Essential features such as interactivity, richness, reliability, and personalization are crucial in influencing user perceptions and behaviors. Interactivity elements, which include real-time feedback and adaptive interfaces, boost user engagement by making interactions more dynamic and responsive [31]. Richness attributes, involving detailed and diverse information provided by map applications, enhance user satisfaction by delivering comprehensive and contextually relevant data [32]. Reliability, characterized by the accuracy and dependability of information, is vital for building user trust, as users depend on these applications for accurate navigation and decision-making [13]. Personalization, which customizes the application experience to meet individual user preferences, further increases satisfaction and loyalty by addressing unique needs [14]. Together, these features cultivate trust and satisfaction, which are essential for the sustained use of map applications [28]. This complex interaction highlights the importance of optimizing these features to enhance the overall user experience and maintain long-term engagement with AI-enhanced map applications.

Compared to traditional paper maps and electronic maps, map apps offer convenient use, timely data updates, a large amount of information, rich functions, and high interactivity [33]. A well-performing map software should be rich in data information, easy to operate, responsive, and accurate in positioning [34]. The reliability, richness characteristics, customization, and interactivity characteristics have been studied in the context of mobile maps [35]. Lee et al. [36] concluded that interactivity characteristics are very important for users' behavior in using travel platforms and classified interactivity into four dimensions: control, bidirectionality, responsiveness, and connectivity. In this paper, after summarizing the characteristics proposed in the above literature, this study proposes that map apps have interactivity characteristics, richness characteristics, reliability characteristics, and personalized characteristics. As intelligent software, the operation mechanism behind map apps is very complex, and users have the right to understand the operation mechanism and algorithm. Based on this, this study explores the influence mechanism of continuance intention based on four characteristics of map apps: interactivity, richness, reliability, and personalization.

### 2.2 Hypotheses developments

#### 2.2.1 Interactivity, satisfaction, and trust

Interactivity within map applications, exemplified by real-time feedback, user engagement, and adaptive interfaces, plays a crucial role in boosting user satisfaction [37]. Research indicates that interactive features enable users to feel more engaged and in control of their navigation experiences, resulting in higher satisfaction levels [38]. For instance, it has been emphasized that interactivity in digital interfaces significantly enhances user experience by fostering more engaging and personalized interactions [39]. Additionally, it has been discovered that interactive elements in mobile applications lead to greater user satisfaction by offering immediate responses and a heightened sense of participation [40]. Consequently, incorporating interactive features such as customizable routes, live traffic updates, and real-time user feedback in map applications can greatly improve user satisfaction [41]. This positive link between interactivity and user satisfaction is well-documented in the literature [42], indicating that interactive features are vital for enhancing overall user contentment in map applications.

The interactivity characteristics reflect the interaction between the user and the technical characteristics of the medium [43]. The impact of interactivity characteristics on satisfaction and trust has been studied. Fiore et al. [44] found that user interaction with website images, which allows users to modify graphic design features, backgrounds, and other similar aspects of website products, significantly contributed to user enjoyment. Websites with strong interactivity characteristics can respond quickly to user behavior and needs, incorporate user comments and suggestions, and make users feel satisfied [45].

Beyond improving satisfaction, interactivity characteristics in map applications are vital for cultivating trust. Trust is essential for users to feel assured of the application's ability to deliver reliable and accurate information [46]. Studies show that interactive features can greatly enhance trust by showcasing the application's responsiveness and dependability [31]. It has been indicated that interactivity builds trust by enabling users to interact with the system in ways that confirm its reliability [47]. Additionally, it has been discovered that higher levels of interactivity increase trust in online platforms, as users view these features as indicators of a well-maintained and user-focused system [48]. By incorporating interactive elements such as real-time assistance, user reviews, and interactive maps, map applications can improve perceived reliability and strengthen user trust [47,49]. This positive relationship between interactivity and trust highlights the importance of designing map applications with interactive features to build and maintain user trust.

According to Animesh et al. [50], interaction performance facilitates users' engagement with the virtual world and provides a sense of enjoyment and immersion. The positive interaction experience that consumers have during their interactions with the merchant increases consumer trust [51]. Clearly, the stronger the interactivity characteristics felt by users in the map app context, the higher the satisfaction and trust they perceive.

According to the analysis of the relationship between interactivity characteristics, satisfaction, and trust, the following hypothesis is proposed in this study.

H1a Interactivity characteristics have a positive and significant effect on map APP user satisfaction.

H1b Interactivity characteristics have a positive and significant effect on map APP user trust.

#### 2.2.2 Richness, satisfaction, and trust

Richness characteristics in map applications, encompassing the depth and variety of information available, are crucial for enhancing user satisfaction [52]. Richness involves the diversity, quality, and comprehensiveness of the content, allowing users to make well-informed decisions [53]. According to Media Richness Theory, richer information media reduces uncertainty and ambiguity, thereby increasing user satisfaction [54,55]. In map applications, richness features such as detailed maps, extensive points of interest, layered information (e.g., traffic conditions, weather updates), and multimedia elements (e.g., images, videos) give users a thorough understanding of their surroundings and navigation options [1]. Research indicates that information richness significantly boosts user satisfaction in online environments by lowering cognitive load and enhancing the perceived value of the service [32,56]. Thus, by incorporating rich and diverse information, map applications can significantly elevate user satisfaction, empowering users and increasing their appreciation for the application's utility and comprehensiveness [57].

As gateways to the mobile Internet, mobile map service providers offer many features to attract users and increase user traffic. Users generally believe that the more features and resources available, the greater the value they derive from mobile maps, which in turn boosts satisfaction with these applications [58]. Some literature also considers functional diversity as a dimension of service quality, considering the importance of functional diversity for mobile maps. In the context of map app usage, richness characteristics are intended to reflect the convenience of having more features and users being able to experience different features. In the context of map app usage, richness characteristics are intended to reflect the convenience of having more features and users being able to experience different features. Further research suggests that the more feature-rich a third-party mobile payment platform is and the more it meets users' needs, the more users will prefer to use it, and their trust in it will increase [59].

Richness characteristics are essential in establishing user trust in map applications [53]. Providing detailed and comprehensive information builds users' confidence in the application's reliability and accuracy. The Information Systems Success Model identifies information quality as a key determinant of user trust [60]. When users perceive the information as rich and trustworthy, they are more inclined to trust the application [61]. Empirical research demonstrated that high-quality and detailed information significantly enhances consumer trust [12]. In the realm of map applications, features like high-resolution maps, detailed route options, real-time updates, and comprehensive location data strengthen users' perceptions of the application's credibility and reliability [62]. This improved perception, in turn, bolsters their trust in the application, as they feel confident that the provided information is accurate and dependable [63]. Thus, the richness of information is a pivotal factor in building and sustaining user trust in map applications.

According to the analysis of the relationship between richness characteristics, satisfaction, and trust, the following hypothesis is proposed in this study.

H2a Richness characteristics have a positive and significant effect on map APP user satisfaction.

H2b Richness characteristics have a positive and significant effect on map APP user trust.

#### 2.2.3 Reliability, satisfaction, and trust

The reliability of map applications, characterized by the accuracy, consistency, and dependability of the information they provide, plays a crucial role in enhancing user satisfaction [64]. Accurate data is essential for users who rely on these applications for navigation and planning [65]. Research underscores that a reliable information system significantly boosts user satisfaction by reducing frustration and enhancing the overall user experience [66]. In the context of map applications, reliability involves providing precise real-time updates, error-free maps, consistent performance, and trustworthy route suggestions. These aspects help users trust the information they receive, leading to higher satisfaction. Moreover, it can be indicated that the quality and reliability of information directly impact user satisfaction by meeting expectations and ensuring a smooth experience [67]. Consequently, when map applications consistently deliver reliable information, users experience greater satisfaction due to reduced cognitive effort and increased confidence in the application's reliability.

Reliability characteristics can be reflected in the following five aspects: whether the company fulfills its promises to customers within the specified timeframe, whether the company is willing to help resolve issues when customers encounter them, whether the company provides quality service from the outset, whether the company completes services on time, and whether the company can offer near-perfect service [68]. Combined with the characteristics of location-based services, the reliability characteristics as the stability of the system and the ability of the service provider to deliver the promised services correctly, timely, and reliably, and empirically demonstrated that the services provided are continuous, stable, and always available, fulfilling the user's relevant service commitments [69,70]. Concerning the above literature, the RELIABILITY characteristics of map APPs aim to reflect the stability of map applications and the ability of service providers to deliver promised services correctly, timely, and reliably.

Reliability features are crucial for developing and sustaining user trust in map applications [71]. Trust is based on the belief that an application will function dependably under various conditions [72]. Furthermore, it can be highlighted that trust in information systems is greatly influenced by their reliability, as users need to be confident that the application will operate correctly and consistently deliver accurate information [73]. In the context of map applications, characteristics such as timely updates, precise location data, and stable performance reinforce user trust by showcasing the application's reliability. Additionally, it was found that the perceived reliability significantly impacted user trust, as reliability is closely linked with the credibility and trustworthiness of the service [74]. Thus, when map applications demonstrate high reliability, they build greater user trust, as users are assured that the application will reliably satisfy their navigation requirements and consistently provide accurate information.

Hadji and Degoulet [75] showed through their study that information resource reliability characteristics affect user satisfaction. Chen and Chou [24] found a positive influence relationship between consumer trust and merchants' ability to provide logistics services reliability characteristics.

According to the analysis of the relationship between reliability characteristics, satisfaction, and trust, the following hypothesis is proposed in this study.

H3a Reliability characteristics have a positive and significant effect on map APP user satisfaction.

H3b Reliability characteristics have a positive and significant effect on map APP user trust.

#### 2.2.4 Personalized characteristics, satisfaction, and trust

Personalized features in map applications, designed to cater to individual preferences and behaviors, play a crucial role in boosting user satisfaction [76]. Personalization entails adjusting content, recommendations, and interface elements to align with the specific needs of users. Studies show that personalization significantly enhances user satisfaction by delivering a more relevant and engaging experience [77,78]. For instance, research discovered that personalized services improve user satisfaction by minimizing information overload and increasing content relevance [79]. In map applications, personalized elements such as tailored route suggestions, location-based recommendations, and user-specific alerts create a more customized and fulfilling user experience. By meeting individual needs and preferences, personalization makes users feel appreciated and understood, leading to higher satisfaction levels [80]. Moreover, it was indicated that personalization boosts usefulness and further enhances satisfaction [81]. Therefore, personalized features in map applications are crucial for making the application more relevant and user-friendly, thereby improving overall user satisfaction.

Personalized characteristics aim to provide humanized services that meet the needs and preferences of each user, emphasizing user value [82]. The advent of the Internet era has changed the original business format, and merchants are increasingly focusing on the user's personality to tailor their services.

Personalized features are also essential in building user trust in map applications [14]. Trust is established when users believe that the application understands and meets their specific needs and preferences [83]. Research suggests that personalization can greatly enhance trust by highlighting the application's focus on delivering user-centric services [84]. In map applications, personalized elements such as customized recommendations, individualized route planning, and user-specific notifications foster trust by demonstrating that the application is attentive and responsive to individual user requirements. Moreover, it has been found that personalization boosts trust by creating a sense of reliability and predictability, as users view personalized services as better aligned with their needs [85]. Additionally, personalizing the user experience can alleviate privacy concerns by clearly showing how user data is used to improve service quality [86]. Thus, personalized features in map applications enhance user trust by offering a more customized and reliable experience, increasing confidence in the application's dependability and purpose.

Xu et al. [87] argue that online stores enhance customer satisfaction by offering services based on individual preferences, shopping history, and specific needs. In the era of mobile internet, product design should prioritize user experience and needs. The success or failure of a product often hinges on whether its details and personalized characteristics satisfy users. Tailoring services to meet individual user needs is a crucial aspect of the mobile internet user experience. Therefore, mobile internet companies should focus on understanding users' special needs, identifying their habits, and improving their products accordingly. Hu et al. [88] verified that user services and personalized characteristics services affect user satisfaction. Yahia et al. [58] explored the factors influencing the formation of consumer trust in the social commerce environment and showed that the security, privacy, and personalized characteristics of websites affect the formation of trust.

According to the analysis of the relationship between personalized characteristics, satisfaction, and trust, the following hypothesis is proposed in this study.

H4a Personalized characteristics have a positive and significant effect on map APP user satisfaction.

H4b Personalized characteristics have a positive and significant effect on map APP user trust.

#### 2.2.5 Satisfaction, trust, and continuous intention

User satisfaction is a vital factor influencing the continuance intention of map application users [30]. Satisfaction represents the overall contentment users feel regarding their experience, which significantly impacts their willingness to keep using the application [89]. Empirical evidence indicates that user satisfaction is a strong predictor of continuance intention in AI-powered service agents contexts [90]. In the case of map applications, satisfaction stems from factors such as ease of use, information accuracy, and the application's overall functionality. When users are pleased with these aspects, they are more likely to develop a positive outlook towards the application, which, in turn, encourages them to continue its use [91,92]. Moreover, it can be indicated that satisfaction fosters loyalty behaviors, including repeated use and recommendations, which are crucial for the ongoing success of digital applications [92,93]. Therefore, improving user satisfaction is essential for maintaining long-term engagement and continuance intention among map application users.

Oliver [94] defines satisfaction as the customer's response to the perceived fulfillment of a product or service, encompassing both the quality of the product and the service itself. This satisfaction level directly correlates with the pleasure or displeasure a consumer experiences, whether meeting, exceeding, or falling short of expectations [95]. Yin and Li [96] found a positive correlation between user satisfaction with mobile apps and intention to continue using them. Lin and Wang [97] found that legal person continuance intention is influenced by user satisfaction.

The level of trust users have in map applications is pivotal for their continued use. Trust indicates the confidence users have in the application's reliability, security, and integrity, which are crucial for ongoing engagement [46]. Trust is fundamental to the adoption and sustained usage of technology [98]. When users have confidence in a map application's dependability for critical activities like navigation and location services, their likelihood of continued use increases [99,100]. Research demonstrated that trust significantly affects users' intentions to persist with online services by lowering perceived risks and uncertainties [101]. In map applications, trust can be nurtured through consistent performance, precise information, and strong privacy safeguards. Trust diminishes feelings of vulnerability, making users feel more secure and committed to long-term use [98]. Hence, establishing and maintaining user trust is essential for encouraging continued use, as trusted applications are more likely to retain users over the long term [102].

Different studies highlight the roles of trust and satisfaction in online continuance intentions across various contexts. McCole et al. [28] constructed a continuance intention model for users of sharing platforms, and the study showed that consumer trust affects users' willingness to continue using.

According to the analysis of the relationship between satisfaction, trust, and continuance intention, the following hypothesis is proposed in this study.

H5 Satisfaction has a positive and significant effect on map APP user continuance intention

H6 Trust has a positive and significant effect on map APP user continuance intention.

With the development of the above hypothetical relationship, this study constructs the theoretical model of map APP user continuance intention, as shown in Fig. 1.

**Fig. 1:** Research framework.

## 3 Research methodology

### 3.1 Research subjects and data collection

AutoNavi Map was selected as the subject of this study. AutoNavi Map is currently the leading provider of digital map content, navigation, and location services in China. With Class A mapping qualifications for navigation electronic maps and Internet map services, its high-quality electronic map database constitutes the core competitiveness of the company. Therefore, selecting AutoNavi Map's users as questionnaire respondents meets the requirements for representativeness in the empirical study. This study used questionnaire research to collect data, so the number and quality of the sample will directly affect the conclusions drawn from the empirical analysis.

AutoNavi Map's user base is diverse, encompassing different ages, geographic locations, usage frequencies, and purposes of use. Stratified random sampling is an effective method to ensure that these distinct groups are well-represented within the sample [103]. This technique involves dividing the population into various subgroups (strata) and then randomly selecting participants from each subgroup. This approach enhances the representativeness of the sample, making it possible to generalize the findings to the entire user population. Given the diverse nature of AutoNavi Map's users, stratified random sampling allows for an accurate representation of different user segments and usage behaviors. This method improves the reliability of the empirical analysis by ensuring that the sample accurately reflects the overall user population's characteristics. By employing stratified random sampling, the study ensures that the collected responses truly represent AutoNavi Map's diverse user base, thus supporting robust and generalizable conclusions.

In this study, the questionnaire was released from the beginning of March 2022 to the end of the questionnaire at the beginning of June 2022, a period of 3 months, 525 questionnaires were collected, and 460 valid questionnaires were retained after eliminating invalid questionnaires.

Specifically, in terms of gender, age, and time of use, each category has a sufficient number of users to be representative of that category of users. The sample size of users with a doctoral degree or above and monthly household consumption expenditure of 10,000 RMB or above is small, which is in line with the current economic income and consumption expenditure, and thus is also representative. This indicates that the data collected by the questionnaire in this study are of sufficient quality and reliability (the details of the sample are shown in Table 1).

**Table 1:** Results for the measurement model.

Construct	Item	Statement	Loading	SMC	α
Interactivity Characteristics	**INC**1	INC1. AutoNavi Map provides an interface for feedback information.	0.791	0.626	0.895
	**INC**2	INC2. I found the AutoNavi Map app to be smooth and lag-free.	0.864	0.746	
	**INC**3	INC3. I can access AutoNavi Map at any time and place to search for information.	0.862	0.743	
	**INC**4	INC4. I feel that AutoNavi Map values my feedback.	0.794	0.630	
Reliability Characteristics	**REC**1	REC1. Steps to complete a task in AutoNavi Map follow a logical sequence.	0.813	0.661	0.906
	**REC**2	REC2. Operating AutoNavi Map always leads to a predicted result.	0.809	0.654	
	**REC**3	REC3. AutoNavi Map responds quickly during the busiest hours.	0.842	0.709	
	**REC**4	RECL4. I think that a quality certification of AutoNavi Map is necessary.	0.810	0.656	
	**REC**5	REL5. I would recommend the use of AutoNavi Map to my colleagues.	0.790	0.624	
Richness Characteristics	RIC1	RIC1. AutoNavi Map's response to the user is very detailed.	0.782	0.612	0.888
	RIC2	RIC2. The information provided by this AutoNavi Map is very clear.	0.849	0.721	
	RIC3	RIC3. AutoNavi Map is expressed in various forms.	0.833	0.694	
	RIC4	RIC4. The amount of information provided by AutoNavi Map is relatively rich.	0.802	0.643	
Personalized Characteristics	**PEC**1	PEC1. AutoNavi Map can predict my preferences and provide targeted services.	0.805	0.648	0.857
	**PEC**2	PEC2. AutoNavi Map can suggest surrounding food, clothing, housing, and transportation based on my usage information.	0.827	0.684	
	**PEC**3	PEC3. AutoNavi Map can provide dialect navigation, celebrity voice navigation, and other special services.	0.816	0.666	
Satisfaction	SAT1	SAT1. I am very content with AutoNavi Map.	0.816	0.666	0.872
	SAT2	SAT2. I am very pleased with AutoNavi Map.	0.837	0.701	
	SAT3	SAT3. I feel delighted with AutoNavi Map.	0.848	0.719	
Trust	TR1	TR1. I'd trust AutoNavi Map to do the work right, even if not monitored.	0.828	0.686	0.878
	TR2	TR2. I trust AutoNavi Map's information to be true.	0.857	0.734	
	TR3	TR3. People (for example, drivers who use AutoNavi Map) on the map app are trustworthy.	0.838	0.702	
Continuance Intention	CI1	CI1. I share the experience of using AutoNavi Map with my friends.	0.783	0.613	0.889
	CI2	CI2. When I have the need, I use AutoNavi Map.	0.864	0.746	
	CI3	CI3. In the future, I will continue to use AutoNavi Map.	0.797	0.635	
	CI4	CI4. I recommend AutoNavi Map to my friends.	0.825	0.681	

Note: SMC= Square Multiple Correlations, Cronbach's alpha = α.

In terms of gender, 282 (61.3 %) were male, and 178 (38.7 %) were female. There are significantly more males than females, mainly because males are more inclined to use map apps compared to females, while females travel relatively less.

Regarding marital status, there were 236 married people and 224 unmarried respondents with a ratio of 51.3 %–48.7 %. In terms of education, there were 154 bachelor's degree holders, 244 master's degree holders, and 62 doctoral degree holders. Among them, 89.1 % were under 30 years old, 8.1 % were between 30 and 50 years old, and 2.8 % were over 50 years old. This distribution aligns well with the actual situation. In terms of consumption level, 141 users (30.7 %) reported a monthly expenditure below 3000 RMB, and 142 users (30.9 %) reported spending between 3000 and 6000 RMB. Users spending between 6000 and 10000 RMB numbered 106 (23 %), ranking second, while users spending over 10000 RMB were the fewest, at 71 (15.4 %). The distribution of continuous usage time was also even, aligning with the actual situation.

### 3.2 Description of research variables

The theoretical model constructed has seven variables, namely, interactivity characteristics, reliability characteristics, richness characteristics, personalized characteristics, satisfaction, trust, and continuance intention. By the paradigm of previous empirical studies, all seven variables were measured in this study by drawing on well-established scales from previous empirical studies.

To be more specific, interactivity characteristics were tested with a four-item scale, which was adapted from Animesh et al. [50]. A 5-item scale proposed by Briz-Ponce et al. [104] and Wu & Zhang [105] was adopted to measure reliability characteristics. 4 items for assessing richness characteristics proposed by Lam et al. [59], 3 items were used to assessment personalized characteristics adopted by Zhang et al. [82]. 3 items for measuring user Satisfaction, which was proposed by Choi [106]. A three-item scale was adapted to assess user trust, which was proposed by Hsu & Lin [107]. A four-item scale was adapted to assess continuance intention, which was developed by Bhattacharjee [108], Thong et al. [109], and Yang et al. [6]. The results of constructs and measures are shown in Table 1. The variables were measured on a seven-point Likert scale, where the items were expressed from 1 to 7 on a scale ranging from "strongly disagree" to "strongly agree".

### 3.3 Analysis method

As in previous Structural Equation Modeling (SEM) data methods, this study uses Amous 24.0 to analyze the collected data [110,111]. As in Wang et al. [112]'s research, the specific process of data analysis in this study is described below. At first, the Confirmatory Factor Analysis (CFA) of the measurement model was examined. The convergent validity of all variables was examined by examining the Standardized Factor Loading, Composite Reliability (C.R.), and Average Variance Extracted (AVE) metrics. Following this, the discriminant validity of the measurement model is examined. The discriminant validity of all the variables is tested by verifying whether there is a difference between the correlations of two different variables. If discriminant validity exists, the structural model is further tested. Immediately after, the model fit of the structural model is tested according to the suggestion of Jackson et al. [113] to determine whether the structural model has a good model fit. If the structural model has a good model fit, it is suitable for further analysis of the research hypotheses. Finally, the hypotheses of this study are tested based on the above analysis to provide theoretical support for the final research conclusions, theoretical contributions, practical insights and future prospects.

## 4 Research results

### 4.1 Assessment of variables

In addition to Cronbach's alpha (see 3.2. Description of research variables), for testing the convergent validity of variables, this study used the composite reliability (C.R.) and the average variance extracted (AVE). To be more specific, the composite reliability of all construct was above 0.857 (interactivity characteristics, 0.897; reliability characteristics, 0.907; richness characteristics, 0.889; personalized characteristics, 0.857; satisfaction, 0.872; trust, 0.879; continuance intention, 0.890), which was over required 0.7, average variance extracted of each construct ranged from 0.840 to 0.922 (interactivity characteristics, 0.686, reliability characteristics, 0.661, richness characteristics, 0.667, personalized characteristics, 0.666, satisfaction, 0.695, trust, 0.707, continuance intention, 0.669) and was above required benchmark value 0.5. These results revealed that the evaluation results were consistent with the benchmark values, thus proving the convergence of the variables.

A further examination of the discriminant validity for all variables was conducted. Examination results revealed that in comparing the correlation between each conformation and the other conformations with the square root of the AVE and the other constructs, the square root of AVE for each variable was greater than the correlations between the variables and the others. These results revealed that the evaluation results were consistent with the benchmark values [114] thus proving the discriminant validity of all variables. Further, this study tested all the measures’ model fit with the Bollen-Stine Bootstrap method to test their model fit. Table 2 presented that the assessment results meet the benchmark value, thus proving the fitting effect of the structural model.

**Table 2:** Results of model fit for structural model.

Fit Indices	Model fit criteria	Measurement model	Results
CFI	>0.9	0.974	Pass
RMSEA	<0.08	0.041	Pass
TLI	>0.9	0.970	Pass
GFI	>0.9	0.943	Pass
NFI	>0.9	0.943	Pass
χ^2^/df	<3	1.785	Pass
AGFI	>0.8	0.925	Pass

### 4.2 Hypothesis testing

Path coefficients analysis was conducted to examine each hypothesized statement (H1∼ H6). Table 3 and Fig. 2 show the final hypotheses testing results.

**Table 3:** Results of regression analyses for hypotheses testing.

Hypothesis	Unstd. Coefficient (β)	S.E.	z-value	Std. coefficient	p-value	Result
INC → SAT	0.162	0.055	2.936	0.180	∗∗	Supported
INC → TR	0.293	0.062	4.747	0.296	∗∗∗	Supported
REC → SAT	0.297	0.057	5.199	0.286	∗∗∗	Supported
REC →TR	0.296	0.063	4.716	0.259	∗∗∗	Supported
RIC → SAT	0.245	0.063	3.911	0.253	∗∗∗	Supported
RIC → TR	0.231	0.069	3.340	0.215	∗∗∗	Supported
PEC → SAT	0.222	0.060	3.673	0.226	∗∗∗	Supported
PEC → TR	0.175	0.066	2.653	0.162	∗∗	Supported
SAT → CI	0.336	0.060	5.637	0.331	∗∗∗	Supported
TR → CI	0.446	0.056	7.940	0.484	∗∗∗	Supported

Note. ∗p < 0.05. ∗∗p < 0.01. ∗∗∗p < 0.001.

Note: Interactivity characteristics = INC, Reliability characteristics = REC, Richness characteristics = RIC, Personalized characteristics = PEC, Satisfaction = SAT, Trust = TR, Continuance intention = CI.

**Fig. 2:** Statistical model diagram.

Consistent with H1a and H1b, the results indicated that interactivity characteristics are positively related to user satisfaction (β = 0.163, p-value <0.01) and interactivity characteristics have a positive and significant impact on user trust (β = 0.293, p-value <0.001). The results of the path coefficients show that both H1a and H1b paths are valid. The results further showed that reliability characteristics are significantly related to user satisfaction and user trust (H2a: β = 0.297, p-value <0.001; H2b: β = 0.296, p-value <0.001)), thereby supporting H2a and H2b paths. Consistent with H3a and H3b, richness characteristics (β = 0.245, p-value <0.001; β = 0.231, p-value <0.001) have a positive and significant impact on user satisfaction and user trust. The results of the path coefficients show that both H3a and H3b paths are valid. The results further showed that personalized characteristics (β = 0.222, p-value <0.001; β = 0.175, p-value <0.01) have a positive and significant impact on satisfaction and trust. The results of the path coefficients show that both H4a and H4b paths are valid. Further, consistent with H5, user satisfaction was also found to be positively related to continuance intention (β = 0.336, p-value <0.01). Thus, H5 was supported. Additionally, the role of user trust was found to have a significant impact on continuance intention (β = 0.446, p-value <0.001). Thus, H6 was also supported.

R-square, or the coefficient of determination, quantifies the extent to which the variance in the dependent variable can be predicted from the independent variables. In this study, the R-square values of continuous intention, trust, and satisfaction were 0.549, 0.641, and 0.656 respectively. In the field of social sciences, which examines human behavior and other intricate interactions, R-square values ranging from 0.50 to 0.70 are typically regarded as satisfactory [115]. Such values indicate that the model accounts for a significant portion of the variance, which is considered acceptable given the inherent unpredictability and complexity associated with social phenomena.

## 5 Discussion

### 5.1 Comparison to other studies

According to the results of the present study, interactivity was significantly associated with satisfaction and trust. This result can be compared to an earlier study by Lee et al. [39]. According to Lee et al.’s [39] study simplicity and interactivity have been identified as key factors influencing mobile phone usability and evaluate their importance through empirical analysis. Additionally, Lee et al.’s [39] research explored how mobile phone usability affected user satisfaction, trust, and brand loyalty. Data for the study was gathered through a survey of mobile phone users. The results of Lee et al.’s [39] research confirmed that simplicity and interactivity are significant determinants of mobile phone usability, with interface simplicity being a crucial prerequisite for a positive interactive and usability experience.

Furthermore, the findings of this study further indicated that reliability had significant associations with satisfaction and trust. The study findings can be compared to an earlier study by Masrek et al. [116]. Masrek et al.’s [116] research was conducted to explore the impact of security and privacy concerns on trust and satisfaction. Additionally, the study aimed to examine how perceived quality affects security, privacy, trust, and satisfaction. Masrek et al.’s [116] research used a survey research method and the study gathered responses from mobile banking users in Malaysia through convenience sampling. The results of Masrek et al.’s [116] research indicated that reliability, encompassing security and privacy, is a significant predictor of trust and satisfaction.

In addition, the present study's findings indicated that richness had a significant relationship with satisfaction. This result can be compared to a study by Gimpel et al. [117]. Gimpel et al.’s [117] research explored the impact of the digital communication channel type and cultural differences between service personnel and customers on customer satisfaction. Gimpel et al. [117] collected data through an online survey simulating a digital service encounter with cultural differences. The findings of Gimpel et al.’s [117] study revealed that richness and social presence significantly affect customer satisfaction.

Moreover, the present study found a significant association between richness and trust. The finding can be somewhat comparable to a study by Chao et al. [118]. The research of Chao et al. [118] explained that with the rise of the internet, virtual communities provide a new avenue for social interaction. Key elements of richness include instant feedback, non-verbal cues, language variety, and personal focus, which are important when considering participation intention. Chao et al.’s [118] research examined the behavior of Facebook users concerning richness characteristics. As users engage in virtual community activities, they encounter various uncertainties. Given these uncertainties, Chao et al.’s [118] study posited that trust is a critical factor influencing participation on Facebook. Chao et al.’s [118] study results indicated that both richness and uncertainty significantly impact participation intention within a virtual community.

In addition, the current study found that personalized characteristics were significantly related to satisfaction and trust. The results can be compared to an earlier study by Carlander et al. [119]. According to Carlander et al. [119], trust is crucial for banks. Carlander et al.’s [119] study explored whether this is true for the relationship between customers and bank employees. The data from Carlander et al.’s [119] study was collected from an online survey of customers of retail banks to create indicator measures. Carlander et al.’s [119] research found that trust in the bank is influenced by the perceived quality of personalized characteristics through employees' perceived competence, benevolence, and transparency. Additionally, Carlander et al. [119] also found that satisfaction with the bank is influenced by the perceived quality of personalized characteristics through perceived competence, benevolence, transparency, and trust.

The present study also indicated a significant relationship between trust and intention to use. The results are somewhat comparable to a study conducted by Rahardja et al. [120]. Rahardja et al.’s [120] research examined the influence of technology mindfulness, technology readiness, and financial literacy on users' intentions to use cryptocurrencies, mediated by perceived trust and perceived risk. Rahardja et al.’s [120] study surveyed individuals who either own cryptocurrencies or have financial investment experience. The findings of Rahardja et al.’s [120] research revealed that perceived trust and perceived risk were found to significantly influence the intention to use cryptocurrencies.

Lastly, the present study found a significant association between satisfaction and intention to use. The results are somewhat similar to an earlier study by Ruangkanjanases et al. [121]. Ruangkanjanases et al.’s [121] research examined how flow experiences influenced the willingness to participate in online purchasing through online shopping platforms. Ruangkanjanases et al.’s [121] study selected internet clients using the convenience sampling technique, and a survey methodology was employed to collect information from internet consumers. Ruangkanjanases et al.’s [121] findings revealed that flow and satisfaction were significantly associated with continuous intention.

### 5.2 Theoretical implications

First, user satisfaction and trust have a positive and significant effect on continuance intention. The results show that the relationship between user satisfaction, trust, and continuance intention is consistent with most studies. After users use the map app for the first time and feel satisfied and trustful, they are likely to continue using the app. In positioning services, the map APP improves the accuracy of positioning. Users have reported that inaccurate positioning sometimes troubles them, making it difficult to judge the direction of travel accurately. For design requirements, the categorization and layout of each function should be clearly delineated, and the interface design should be simple, clear, and prominently feature core functions. Therefore, the accurate positioning of the map app, simple interface design, and easy-to-use functions are hypothesized to enhance users' satisfaction and trust, thereby positively influencing their continuance intention.

Second, there is a positive influence of the interactivity characteristics, richness characteristics, reliability characteristics, and personalized characteristics of map apps on user satisfaction. With the improvement of people's living standards and lifestyles, map apps not only provide voice navigation and information recommendations but also personalized services that can better meet users' diversified needs and enhance market competitiveness. From a technical aspect, the map app improves user satisfaction by enhancing the smoothness of software operations. For example, real-time changes in road information during user travel require a smooth operation to avoid missing the best route. Thus, it is hypothesized that the virtual technology of the map app enhances users' interactivity, richness, reliability, and personalized characteristics, thereby positively affecting their satisfaction.

Third, the interactivity characteristics, reliability characteristics, richness characteristics, and personalized characteristics of the map app significantly and positively affect users' trust. This may be due to the open operation mechanism of map app software operators. The higher the degree of specialization, the more users can understand or judge whether their privacy and property are at risk. The geographic information and functions provided by map apps effectively meet people's daily life and travel needs, influencing their perception and trust in the app. Consequently, residents may choose to use other apps with similar functions as alternatives to meet their needs.

Hence, to summarize the theoretical implications. The frequent incorporation and importance of both trust and satisfaction underscore the relevance of these additional variables like interactivity, reliability, richness, and personalized characteristics in comprehending the factors that influence user acceptance of Apps. Moreover, the impact of trust and satisfaction across various industries and demographics highlights their adaptability and underscores their significance in the extended Technology Acceptance Model (TAM). Therefore, it can be argued that while traditional base theories are important, unique factors such as trust and satisfaction must be considered to fully understand user acceptance. Consequently, it is advised that future research should expand traditional acceptance models to include trust and other attitude-related constructs. This insight is crucial for the advancement of theoretical frameworks.

### 5.3 Practical implications

First, map APP operators should continuously innovate mobile map application technology, introduce new functions and services that meet users' needs, update and improve geographical information promptly, and supplement with text or video descriptions to mobilize users' enthusiasm to use and increase their understanding of the operation mechanism. At the same time, operators should pay attention to both the user's needs for applications and products' personalized characteristics. For example, users can make more personalized settings for the map APP according to their usage preferences to enhance their experience [122], pay attention to users' experience of interactivity characteristics in the map APP, and establish corresponding community sections for users to communicate their purposes and find entertainment and food near them to enhance their sense of participation.

Second, map APP operators should not only pay attention to the authenticity, timeliness, and credibility of the information provided to ensure that the relevant information users get real and valid but also focus on considering the technical applications of map APP in data mining, image recognition and deep learning to plan scientific and reasonable travel routes for users and solve problems such as difficulties in user positioning. Meanwhile, map APP as a smartphone application, operators should focus on the stability of the map APP port, connection speed, and privacy protection when developing and designing to improve the reliability of the map APP. In addition, operators should establish a sound information feedback mechanism to ensure that users can get timely feedback on the problems they respond to customer service.

Third, due to the fierce competition in the map APP market, it is not enough to rely on operators to optimize and upgrade map APPs to promote users' continuous use, and the government should also formulate corresponding industry regulations and incentive laws and regulations. For example, the map market is strictly forbidden to attract users' use through malicious competition, such as encouraging businesses and enterprises to enter map-based APPs. In addition, the government should also encourage the companies in the map-based APP market to develop together in competition and cooperation.

Hence, to summarize the practical implications of this research. Boosting interactivity and richness in AI applications can significantly enhance user satisfaction by making them more engaging and informative [123]. Developers should focus on designing dynamic interfaces and offering comprehensive, contextually relevant content to elevate the user experience. Furthermore, maintaining the reliability of AI applications is essential for fostering and sustaining user trust. This can be accomplished by delivering accurate and consistent information, and by demonstrating the application's reliability. Personalization is also crucial for building trust and satisfaction, indicating that AI applications should be customized to suit individual user preferences and needs. By emphasizing these characteristics, businesses can increase user acceptance and promote the continuous use of AI applications. Additionally, these findings can guide the creation of targeted marketing strategies that emphasize the interactive, reliable, and personalized features of AI applications, thus attracting and retaining users [124].

### 5.4 Research limitations and future research development

First, this study provides empirical evidence on mobile map app usage in the context of mobile internet research, relying primarily on online questionnaires for data collection. However, this single-source data approach may limit the study's scope. Future research could enhance validity by diversifying data sources and capturing a broader range of respondents, thereby ensuring findings are more representative and generalizable.

Second, the theoretical model constructed in this study mainly considers the effects of interactivity characteristics, reliability characteristics, richness characteristics, and personalized characteristics on intention to use and does not consider other dimensions of factors that affect mobile map users not included in the model. Therefore, future research can include other dimensions (for instance, brand image [125], big data analytics [2,126], and artificial intelligence [127]) in the research model, including the mediating and moderating roles, to further enrich the theoretical model of user Continuance Intention of the map APP.

Third, little research has been conducted on the specific types of map APP user Continuance Intention. Therefore, based on the study of map APP user Continuance Intention, this study can go further and consider the differences in user behavior that may be caused by the differences between different types of map APPs. To explore the factors influencing the Continuance Intention of different types of map APP users and their mechanisms in the process of achieving the integration of the map industry and Internet industry.

## 6 Conclusion

This study examined how interactivity, richness, reliability, and personalization affect user satisfaction and trust in AI-driven map applications, and how these factors influence users' intention to continue using these applications. The results highlight the important role these characteristics play in shaping user experience. Interactivity and richness improve user satisfaction by delivering engaging and comprehensive content, while reliability and personalization build trust through accurate, consistent, and user-focused information. These findings enhance the theoretical understanding of the impact of specific application features on user behavior within AI-enhanced services. For developers and operators of map applications, focusing on these characteristics can boost user satisfaction and trust, which are crucial for long-term user engagement. By improving interactivity, ensuring rich information, maintaining reliability, and personalizing user experiences, map application providers can better meet user expectations and encourage ongoing use. Additionally, this study fills a gap in the literature by providing empirical evidence on the factors driving continuance intention in AI-driven map applications, offering a detailed understanding of user behavior in this area.

## CRediT authorship contribution statement

**Athapol Ruangkanjanases:** Writing – review & editing, Writing – original draft, Methodology, Formal analysis, Data curation, Conceptualization. **Ornlatcha Sivarak:** Writing – review & editing, Writing – original draft, Methodology, Formal analysis, Data curation, Conceptualization. **Chin-Tsu Chen:** Writing – review & editing, Writing – original draft, Methodology, Formal analysis, Data curation, Conceptualization. **Asif Khan:** Writing – review & editing, Writing – original draft, Methodology, Formal analysis. **Shih-Chih Chen:** Writing – review & editing, Writing – original draft, Methodology, Formal analysis, Data curation.

## Availability of data and materials

Data will be provided on reasonable request from the corresponding author.

## Ethics approval (non-biological or non-medical manuscripts do not need to write this part)

Not Applicable.

## Funding statement

Not Applicable.

## Declaration of competing interest

The authors declare that they have no known competing financial interests or personal relationships that could have appeared to influence the work reported in this paper.
